The article "Multiple Sclerosis: The Role of Cytokines in Pathogenesis and in Therapies" was retracted in 2016. Reasons: plagiarized text; overlap with other authors' work.

# Multiple Sclerosis: The Role of Cytokines in Pathogenesis and in Therapies

**DOI:** 10.3390/ijms131013438

**Published:** 2012-10-19

**Authors:** Amedeo Amedei, Domenico Prisco, Mario Milco D’Elios

**Affiliations:** 1 Department of Internal Medicine, University of Florence, Largo Brambilla 3, Florence 50134, Italy; E-Mail: delios@unifi.it; 2 Department of Biomedicine, Patologia Medica Unit, Azienda Ospedaliero-Universitaria Careggi, Largo Brambilla 3, Firenze 20134, Italy; E-Mail: priscod@aou-careggi.toscana.it; 3 Center of Oncologic Minimally Invasive Surgery, University of Florence, Largo Brambilla 3, Florence 50134, Italy; 4 Department of Medical and Surgical Critical Care, University of Florence, Largo Brambilla 3, Florence 50134, Italy

**Keywords:** multiple sclerosis, cytokines, T helper cells (Th), Interleukin-17 (IL-17), Interferons (IFNs)

## Abstract

Multiple sclerosis, the clinical features and pathological correlate for which were first described by Charcot, is a chronic neuroinflammatory disease with unknown etiology and variable clinical evolution. Although neuroinflammation is a descriptive denominator in multiple sclerosis based on histopathological observations, namely the penetration of leukocytes into the central nervous system, the clinical symptoms of relapses, remissions and progressive paralysis are the result of losses of myelin and neurons. In the absence of etiological factors as targets for prevention and therapy, the definition of molecular mechanisms that form the basis of inflammation, demyelination and toxicity for neurons have led to a number of treatments that slow down disease progression in specific patient cohorts, but that do not cure the disease. Current therapies are directed to block the immune processes, both innate and adaptive, that are associated with multiple sclerosis. In this review, we analyze the role of cytokines in the multiple sclerosis pathogenesis and current/future use of them in treatments of multiple sclerosis.

## 1. Introduction

Multiple sclerosis (MS), the clinical features and pathological correlate for which were first described by Charcot, is a chronic neuroinflammatory disease with unknown etiology and variable clinical evolution. Because the neuroinflammatory process usually starts in patients in their early twenties, some authors hypothesized a slow infection during adolescence as a possible (co)factor of MS. Many viruses have been suspected and studied in this regard, but so far no specific virus has been found to be the MS cause [1,2]. Finally, one of the current MS treatments is with IFN-which was originally discovered as a broad spectrum antiviral agent [3,4].

Multiple sclerosis strikes twice as many women than men and worldwide, about 2–3 million MS patients are mainly found in Europe and in countries with Caucasian immigration, such as USA, Australia and Northern Asia [5,6]. The possible influence of the geographic environment has been studied using monozygotic twins that obtain the MS prevalence from their prepubertal geographic destination [7].

Although neuroinflammation is a descriptive denominator in MS based on histopathological observations, namely the penetration of leukocytes into the central nervous system (CNS), the clinical symptoms of relapses, remissions and progressive paralysis are the result of losses of myelin and neurons [8,9]. In analogy with other multifactorial diseases, MS is influenced by genetic and environmental factors. Therefore, in the absence of etiological factors as targets for prevention and therapy, the definition of molecular mechanisms that form the basis of inflammation, demyelination and toxicity for neurons have led to a number of treatments that slow down disease progression in specific patient cohorts, but that do not cure the disease.

The perfect MS drug should reverse the processes of neuroinflammation, demyelination and neuronal loss, but such substances do not exist. Therapies have been refined beyond anti-inflammatory glucocorticosteroids.

The introduction of IFN-, copolymer and, more recently, natalizumab, monoclonal antibody (Moab) against a1b4 integrin, has considerably improved the life of many MS patients, But intrinsic therapeutic limitations and severe side effects associated with these drugs, stimulate basic and clinical researchers to define innovative and more patient-compliant treatment strategies.

With the latest tools of molecular biology, such as whole genome sequencing, genome-wide association studies [10,11], gene expression profiling coupled with protein analysis [12,13], we may be able, in the future, to define common identifiers for specific cohorts of MS patients, to perform better and earlier diagnoses and, hopefully, discover etiological factors.

However, this is presently not yet possible and therapies are directed to block the immune processes, both innate and adaptive, that are associated with MS. In this review we analyze the role of cytokines in the MS pathogenesis and current/future use of them in treatments of multiple sclerosis.

## 2. The Role of T Cells-Associated Cytokines in MS Pathogenesis

About 15 years ago, Opdenakker and colleagues assembled the available information from histopathological data and inflammation-associated components to create the REGA (Remnant Epitopes Generate Autoimmunity) model to understand MS and to place MS therapies into a new context. In this model, the proteinases, notably matrix metalloproteinases (MMP), cleave substrate proteins into autoimmune peptides that (re)activate specific T cells [14] (Figure 1).

The model used MMP-2 and MMP-9 as examples of proteinases, because previous publications linked MMP-9 in the cerebrospinal fluid with multiple sclerosis and other neuroinflammatory diseases and because myelin basic protein (MBP) was cleaved into immune-dominant peptides by MMP-9 [15,16]. Although most recognized for these two aspects, the REGA model contained much more information related to autoimmune diseases (e.g., about regulatory cytokines) that was instrumental and will remain important for the future drug development [14]: (a) it addressed the critical point that (unspecific) inflammatory reactions with myeloid cells may be primordial and a possible target in MS. In 1994, this was rather controversial and led to some opposition in an era when most MS research was centered on T cells. (b) It translated the central stage of inflammation in the autoimmune process into molecules and addressed the importance of balances between pro-inflammatory versus anti-inflammatory primary cytokines in the disease process. Interleukin-1β (IL-1β), TNFα (Tumor Necrosis Factor-α) and IFN-γ (Interferon-γ) were included as pro-inflammatory cytokines and IFN-α/β and TGF-β (Transforming growth factor β) as anti-inflammatory cytokines. (c) It addressed the role of myeloid antigen presenting cells in the activation of T cells. Moreover, MBP-specific T cells isolated from MS patients and encephalitogenic T cells recovered from immunized animals have confirmed that T cells play a central role in the MS pathology [17–19].

EAE (Experimental Autoimmune Encephalomyelitis), the most studied MS animal model, is an acute or chronic-relapsing, acquired, inflammatory and demyelinating autoimmune disease. The animals are injected with the whole or parts of various proteins that make up myelin. These proteins induce an autoimmune response in the animals—that is, the animal’s immune system mounts an attack on its own myelin as a result of exposure to the injection. The animals develop a disease process that closely resembles MS in humans. EAE has been induced in a number of different animal species including mice, rats, guinea pigs, rabbits, macaques, rhesus monkeys and marmosets. For various reasons including the number of immunological tools, the availability, lifespan and fecundity of the animals and the resemblance of the induced disease to MS, mice and rats are the most commonly used species. The animals are inbred to reliably produce susceptibility to EAE in the animals. As with humans and MS, not all mice or rats will have a natural propensity to acquire EAE. Moreover, different breeds will develop different forms of EAE, some of which act as good models for the different human forms of MS. Different EAE forms are also used as models for the different stages of MS. Even though EAE is the best MS model, it is not multiple sclerosis and a number of significant assumptions are made when proposing EAE as an animal model for MS. Several proteins or parts of proteins (antigens) are used to induce EAE including: Myelin Basic Protein (MBP), Proteolipid Protein (PLP), and Myelin Oligodendrocyte Glycoprotein (MOG), but, importantly, EAE can also be induced by adoptively transferring an expanded population of myelin-specific encephalitogenic CD4+ (T helper (Th)) cells [20], precisely, selfreactive Th1 clones [21].

In the 1990s, Mosmann and Coffman postulated that Th cells can be classified into two distinct subsets, Th1 and Th2. Th1 cells produce large quantities of IFN-γ, driven by IL-12, which promotes cellular immunity directed against intracellular pathogens. Alternatively, Th2 cells, which secrete IL-4, IL-5, IL-13, and IL-25, are essential in the destruction of extracellular parasites and the mediation of humoral immunity [22,23].

Increased levels of Th1 cytokines are particularly evident during EAE/MS relapse, whereas increased Th2 cytokines are found during remission in MS patients [24]. Clinical and hematological symptoms are exacerbated in relapsing/remitting MS patients following the IFN-γ administration, and this is also observed in other Th1-type diseases, whereas it is less apparent in Th2 diseases [25,26]. In other words, Th1 cells were earlier thought to be pathogenic T cells, whereas Th2 cells were thought to confer an anti-inflammatory potential, constituting protective T cells in both MS and EAE [27–30].

However, this clear-cut immune-dysregulation of the Th1/Th2 balance in EAE and MS may be part of a hidden complex of interactions underlying EAE and MS [31]. The Th1-driven nature of the MS disease was challenged by the discovery that IFN-γ and IFN-γ-receptor-deficient mice, as well as mice that lack other molecules involved in Th1 differentiation, such as IL-12p35, IL-12 receptor β2 (IL-12Rβ2, and IL-18, were not protected from EAE, but instead were more susceptible to the disease [32–36]. Unexpectedly, mice deficient in IL-12α (IL12p35, a component of the Th1 paradigm, are vulnerable to EAE. Similarly, IL-12Rβ2-deficient mice develop more severe clinical manifestations of EAE, whereas IL-12p40-deficient mice are resistant to EAE [34,35,37]. These contradictory data indicate that an imbalance in the Th1/Th2 milieu cannot explain the overall immunopathogenic mechanisms underlying multiple sclerosis.

### 2.1. Immunopathogenic Function of IL-17

When the p19 (a novel cytokine heavy-chain homolog of the IL-6 subfamily) chain is linked to the p40 chain, a subunit of IL-12 (another IL-12 subunit is the p35 chain), it forms a novel cytokine designated IL-23. Cua and colleagues verified that IL-23, but not IL-12, is essential for the induction of EAE by generating IL-23p19 knockout (KO) mice and comparing them with IL-12p35 KO mice [38]. Furthermore, an IL-17-producing T cell subset, driven and expanded by IL-23, can pathogenically induce EAE when adoptively transferred into naive mice [39,40]. These IL17-producing T cells were dramatically reduced in the CNS of IL-23p19-deficient mice. These results suggested that IL-17-producing CD4^+^ T cells are a distinct and novel Th subset that exacerbates autoimmunity, and designated them Th17 cells [41,42].

The Th17 discovery further clarifies the cytokine MS profile [43] and, recently, the levels of IL-17 produced by MBP-stimulated peripheral blood cells were shown to correlate with the active lesions in MS patients [44].

Like other Th subsets, the Th17 lineage is activated by a specific cytokine milieu. However, IL-23 cannot produce Th17 cells de novo from naïve T cells, and the IL-23 receptor (IL-23R) is not expressed on naïve T cells [45].

TGF-β up-regulates IL-23R expression, thereby conferring responsiveness to IL-23. These data confirm that TGF-β is a key cytokine in the commitment to Th17 expansion [46]. In mice, TGF-β together with IL-6 can activate antigen-responsive naïve CD4^+^ T cells to develop into Th17 cells [47].

In humans, naïve CD4^+^ cells exposed to IL-6, TGF-β, and IL-21 can develop into Th17 cells; and the IL-23 production plays a role in maintaining these Th17 cells [48,49]. Altogether, Th17 cells require IL-23, TGF-β, IL-6, and IL-1 for their generation.

Th17 cells produce IL-17 (A and F), which are upregulated in chronic lesions [50,51], and IL-22, which is also involved in the MS pathogenesis. Also, microarray studies of lesions in MS patients demonstrated an increased IL-17 expression, confirming that Th17 cells play an important role in the development of inflammation and damage of the CNS.

Patients with MS have greater numbers of IL-17-mRNA-expressing mononuclear cells in the cerebrospinal fluid (CSF) than in the blood. Previously, no increase in the numbers and expression of IL-17 mRNA by mononuclear cells isolated from the CSF was observed in MS patients, but higher levels of IL-17 mRNA were observed in the CSF than in the blood, with the highest levels in the blood detected during clinical exacerbations [52]. These data confirm the pivotal role of IL-17 in MS both peripherally and centrally.

### 2.2. Reciprocal Interactions of Cytokines Produced by T Cells

IL-1R KO mice have impaired Th17 cells and are protected from EAE [53]; also, IL-1β increases the progression of relapse onset in MS [54], implying a role for IL-1β in the development of EAE and MS. EAE was abolished by a virus-expressing IL-4 but not IL-10 in chronic relapsing EAE. Therefore, the cytokine environment was converted from a disease-promoting IL-23-producing condition to a disease-limiting IL-4-producing condition by the local expression of IL-4 from a Herpes simplex virus vector delivered to the brain [55]. Moreover, the increased expression of IL-4 in glial cells was associated with the reduced EAE severity [56], suggesting that the upregulation of Th2 cytokines inhibits the propagation of the EAE/MS inflammation promoted by Th17.

TGF-β is a key cytokine in the generation of the regulatory T cells (Tregs), that inhibit the autoimmune response and protect against inflammatory injury. Tregs are involved in the regulation of Th1/Th2 and Th17 cells. Therefore, the generation of pathogenic Th17 cells induce autoimmunity, the generation of Tregs inhibit autoimmune tissue injury [57].

Although EAE was once considered a classical Th1 disease, it has been proposed that it is predominantly Th17 driven. The data about IL-17 and IFN-γ in MS genesis, indicate that their roles may depend on the nature of the immune response and that the IL-17 may overcome the inhibitory effect of IFN-γ, which generally prevents inflammation at the brain [58].

When pure Th17 cells, polarized with TGF-β to deplete any IFN-γ production, are adoptively transferred to mice, they do not induce EAE, suggesting that the reciprocal interactions among Th17-related cytokines enroll and activate the involvement of associated immune cells. Interestingly, when Th17 cells are combined with Th1 cells, they can fully induce EAE disease [59]. Liu and colleagues also demonstrated that the loss of STAT3 by T cells results in an intrinsic developmental defect that renders STAT3−/− mice resistant to CNS inflammatory diseases. STAT3 is required for the production of IL-17 by Th17 cells, the generation of double positive T cells expressing IL-17 and IFN-γ, and T cell trafficking into CNS tissues. This suggests that STAT3 may be a therapeutic target for modulating CNS autoimmune diseases [60].

A recent study showed significant differences in the regulation of inflammation in the brain and spinal cord, depending on different Th17/Th1 ratios, by demonstrating that specific T-cell populations targeting different myelin epitopes are characterized by different Th17/Th1 ratios in EAE [61]. Also, the Th1 have the potential to reciprocally regulate Th17 cells during EAE.

IL-21 is a type I four-α-helix bundle cytokine that belongs to the IL-2 family and functions as a “growth hormone”—like cytokine. In detail, IL-21 plays a pivotal role in the expansion and differentiation of the Th17 lineage [62]. During clonal expansion, IL-21 also promotes IL-23R expression in differentiated Th17 cells, which plays an important role in the stabilization of the Th17 lineage in the presence of IL-23 [63]. Although no effects were observed when IL-21 was administered after EAE progression, the IL-21 administration boosted natural killer (NK) cell functions before the induction of EAE, including the secretion of IFN-γ [64].

Alternatively, IL-27 (an IL12/IL23 family member) is a negative regulator of Th17 cell differentiation and can prevent inflammatory demyelination in the EAE model [65].

IL-27 drives the expansion and differentiation of IL-10-producing Tregs by inducing the expression of three key molecules: the basic leucine-zipper transcription factor Maf (generally known as c-Maf), the IL-21, and ICOS (an inducible T**-**cell costimulator structurally and functionally related to CD28. Moreover, IL-27-driven c-MAF expression transactivates the production of IL-21, which favor the expansion of IL-27-induced Tr1 cells. ICOS also promotes IL-27-driven Tregs. Each of these elements is essential, because the loss of c-MAF, IL-21 signaling, or ICOS reduces the frequency of IL-27-induced Treg differentiation (Figure 2) [66]. Exacerbation of EAE was demonstrated in IL-27-deficient mice, and interestingly, IL-27 treated mice had markedly reduced CNS inflammatory infiltration, indicating the downregulation of Th17 phenomena [67].

Recently, a novel effector T-cell subset, Th9 cells, has been identified, and the ability of this T-cell subset to induce EAE is currently being investigated. Jager and colleagues generated specific Th17, Th1, Th2, and Th9 cells *in vitro* to directly characterize their encephalitogenic potency after adoptive transfer. They found that Th1, Th17, and Th9 cells, but not Th2 cells, induce EAE. Interestingly, each T-cell subset induced disease in a distinct pathological manner, suggesting that the different effector Th subsets that induce EAE do so differently and implying that the pathological heterogeneity in MS lesions might be partly attributable to various characteristics of myelinreactive effector T cells [68,69]. The authors also suggested that MS might be a disease caused by multiple distinct myelinreactive effector cells. The disease induced by Th17 cells in some animals exhibited symptoms atypical of EAE, including ataxia, severe imbalance, and weight loss associated with high mortality. Some animals had a mixture of atypical and typical EAE symptoms. When cells were recovered from the CNS, it appeared that the transferred Th9 cells produced IFN-γ. The identities of the other cell populations did not seem to drift after their *in vivo* transfer [69].

It has recently been demonstrated that cultured in the presence of TGF-β, Th17 cells produce IL-9. Th17 cells generated *in vitro* with IL-6 and TGF-β and *ex vivo*-purified Th17 cells both produced IL-9. Also, the IL-9 neutralization and IL-9R deficiency attenuated the disease, and this correlated with reductions in Th17 cells and IL-6-producing macrophages in the CNS. These data confirmed the IL-9 role in the EAE development/progression and suggested IL-9 as a Th17-derived cytokine that contributes to inflammatory disease [70].

## 3. Cytokines and Innate Immune Cells in MS

Myelin is presented in the circulation, and other CNS antigens are thought to be expressed in the cervical lymph nodes, which can trigger the conversion of myelin-specific T cells to pathogenic T cells. Adhesion molecules, the integrins, allow these myelin-specific T cells to penetrate the blood–brain barrier (BBB) under inflammatory conditions, and in this way, activated and memory T cells can enter the CNS [71]. Myelin-specific T cells migrate into the CNS and the movement of antigen-presenting cells (APCs) into the CNS is essential for lymphocyte reactivation and the initiation of the inflammatory cascade in the EAE development [72]. Subsequently, inflammatory and immune cells, such as granulocytes and macrophages, are attracted into the CNS parenchyma, where they mediate tissue inflammation and tissue damage [73].

The brain was formerly considered an immune-privileged organ, but today, we understand that any damage to the CNS can activate immune cells *in situ*, particularly microglial cells, that have a key role in maintaining the autoimmune responses in the CNS [74].

Also, microglial cells upregulate the expression of MHC (major histocompatibility complex) and costimulatory molecules to initiate the generation of the inflammatory milieu. Dendritic cells (DCs) seem to play a critical role in antigen presentation to invading T cells and in the of cytokines/chemokines release, thereby guiding into the lesion the entry of monocytes and lymphocytes [75].

Whereas the CD4^+^ cells recruit macrophages, which release proinflammatory cytokines (IL-1, IL-6, TNF-α), destructive molecules (nitric oxide) and MMPs, the CD8^+^ T cells directly attack MHC class I-expressing cells (oligodendrocytes and neurons) [76,77]. TNF receptor 1 (TNFR1 but not TNFR2 signaling is critical for demyelination and the limitation of T-cell responses during immune-mediated CNS disease [78]. This complicated process triggers the recruitment of innate immune cells, especially macrophages and microglia, which in turn mediate demyelination, axonal damage, and lesions.

In autopsy samples from MS patients, the expression of IL-17 is evident in perivascular lymphocytes and in astrocytes and oligodendrocytes located in the active areas of CNS lesions.

IL-17R is also identifiable in acute and chronic plaques of MS patients, suggesting the enrichment of Th17 and CD8^+^ T cells in active MS lesions [79]. Also, microarray analysis of MS lesions has demonstrated increased transcripts of genes encoding inflammatory cytokines, particularly IL-6, IL-17, and IFN-γ. A significant increase in IL-23 mRNA and protein expression is found in lesion tissues and activated macrophages, microglia and especially mature DCs have been shown to be important sources of IL-23p19 [80].

There is also evidence that MS endothelial cells express high levels of IL-17R and are more permeable to IL-17. This microenvironment favors the differentiation of naïve CD4^+^ T cells into Th17 cells, that transmigrate efficiently across BBB endothelial cells (BBB-ECs), leading to the destruction of human neurons and initiating CNS inflammation [81]. Similarly, the expression of IL-17R and IL-22R on BBBECs has been examined in MS lesions, and IL17 and IL-22 have been shown to disrupt BBB tight junctions *in vitro* and *in vivo*. IL-6 transsignaling may also play a role in the autoimmune inflammation of the CNS, mainly by regulating the early expression of adhesion molecules, possibly via cellular networks at the BBB [82]. Ifergan and colleagues demonstrated that a subset of monocytes migrate across the inflamed human BBB and differentiate into DCs under the influence of BBB-secreted TGF-β and GM-CSF (granulocyte macrophage colony-stimulating factor). These DCs can produce IL-12p70, TGF-β, and IL-6 and promote the expansion of Th1 and Th17 cells. The abundance of such DCs *in situ* is strongly associated with microvascular BBB-ECs within acute MS lesions and with a significant number of Th17 cells in the perivascular infiltrate [83].

Astrocytes play significant physiological roles in CNS homeostasis and act as a bridge between the CNS and the immune system. Astrocytes also contribute to the complex interactions during CNS inflammation. IL-17 functions in a synergistic manner with IL-6 to induce IL-6 expression in astrocytes. Astrocytes upregulate the expression of IL-17 and IFN-γ in T cells, which is consistent with the capacity of astrocytes to express IL-23 subunit p19 and the common IL12/IL23 subunit p40, but not IL-12 subunit p35 [84]. Recently, increased IL-17RA expression in the CNS of mice with EAE and in both astrocytes and microglia *in vitro* [85] has been demonstrated.

Also, the suppressor of cytokine signaling 3 (Socs3 participates in IL-17 functions in the CNS as a negative feedback regulator, in fact mouse models of Socs3 small interfering RNA (siRNA) knockdown and Socs3 deletion, showed enhanced IL-17 and IL-6 signaling in astrocytes, indicating that astrocytes can act as a target of Th17 cells and IL-17 in the CNS [86]. Similarly, in mice deficient of Act1, critical for IL17 signaling, the Th17 cells showed normal infiltration into the CNS but failed to recruit lymphocytes, neutrophils and macrophages. Therefore, astrocytes are critical in IL-17–Act1-mediated leukocyte recruitment during EAE [87].

Interestingly, the data obtained by a monkey MS model established that macrophages respond to the Th1 milieu and neutrophils respond to Th17 cytokines. Also, the study showed dense accumulations of T/B cells and macrophages/microglia at the sites of perivascular and parenchymal lesions in the neocortex and subcortical white matter, indicating that the inflammatory response, especially activation of macrophages and microglia, may be regulated differently in the gray matter areas of the primate brain [88].

In summary, DC-like cells in the peripheral tissues and microglia in the CNS are responsible for cytokine polarization and the Th17 expansion. The complex interactions of Th17 cells with different cells, such as y microglia, astrocytes, neutrophils and macrophages, all contribute to the MS immunopathogenesis.

## 4. Current and Future Clinical Applications of Cytokine-Mediated Treatments

Our understanding of the MS patho-physiology has led to the development of novel therapeutic strategies. Since the early 1990s, disease-modifying drugs have been introduced for the selective MS management, including IFN-β and glatiramer acetate (GA), which have become the standard treatment for relapsing/remitting MS [89] but in this paragraph we analyze, in detail, three domains of novel immune-mediated therapeutics used for MS; the first domain includes immunosuppressive/immunomodulator agents, such as mitoxantrone, laquinimod (ABR-215062, cladribine (Mylinax), and teriflunomide. The second domain includes immune-modulatory agents: (a) cytokine inhibitors such as IFN-β; (b) agents that deplete specific immune cell subsets, such as alemtuzumab (a human mAb targeting CD52 expressed especially by T cells) [90,91] and rituximab (which targets CD20 to deplete B cells) [90,92]; (c) agents that selectively block coreceptors and costimulators, such as daclizumab (an anti-CD25 mAb that inhibits activated T cells and induces regulatory immune cells) [93]. The third domain includes neuroprotective agents associated with immunomodulation, including broad-spectrum immunomodulators such as statins, PPAR agonists (e.g., pioglitazone, gemfibrozil), the sex hormone estriol (E3, fumarate and minocycline), all of which have been effective in the MS treatment.

IFN-β has been clinically introduced to treat MS patients based on its ability to shift a Th1-mediated response to a Th2 phenotype. However, microarray studies have indicated that a number of genes in MS patients are upregulated by the cytokines associated with the differentiation of T cells into Th1 rather than into Th2, suggesting that this shift may not be the only therapeutic mechanism of IFN-β in MS [94]. IFN-β therapy also reduces IL-23 mRNA levels [95] and inhibits human Th17 cell differentiation, so the Th17 axis could be another target of IFN-β therapy [96]. IFN-β-mediated IL-27 production by innate immune cells has been shown to play a critical role inhibiting Th17 cells in [97]. In addition, the therapeutic effect of IFN-β is probably attributable to the induction of the regulatory cytokine IL-10 [95]. A high IL-17F level in the serum of people with relapsing/remitting MS is associated with the failure of IFN-β therapy. This characteristic of IFN-β might contribute to an exploration of some logical biomarkers for predictive assessment of the response to a popular therapy for MS [98].

IFN-β inhibits the Th17 expansion in MS, and this might contribute to an improvement in the clinical symptoms. The effectiveness of this inhibition, however, requires intact IFN-γ signaling in T cells. In a recent study, Conti and colleagues reported that both mRNA and cell surface expression of the signaling chain of the IFN-γ receptor (IFN-γR2 and its cognate tyrosine kinase JAK2 are enhanced in peripheral blood Th17 cells and clones from patients with active MS compared with those with inactive MS. IFN-γ decreased the frequency of Th17 peripheral cells and proliferation of Th17 clones from patients with active MS; also the stimulation of healthy donors PBMCs in Th17-polarizing conditions resulted in the enhancement of JAK2 expression and accumulation of cell surface IFN-γR2. The role of JAK2 in the modulation of IFN-γR2 was demonstrated as its transduction prevented rapid internalization and degradation of IFN-γR2 in JAK2-deficient γ2A cells. In others words, these data identify JAK2 as a critical factor that stabilizes IFN-γR2 surface expression in Th17 cells from patients with active MS, making them sensitive to IFN-γ [99].

Although B cells may have a dual role in the pathogenesis of MS, they contribute to the induction of the autoimmune response but also mediate the resolution of the CNS inflammatory infiltrate [100,101]. A recent study demonstrated that supernatants transferred from IFN-β-treated B cells inhibited Th17 cell differentiation and suppressed the secretion of IL-17A. Likewise, IFN-β also induces in B cells the IL-10 secretion which may mediate their regulatory potency [102]. Thus, IFN-β exerts its therapeutic effects at least in part by targeting B cells’ functions that contribute to the autoimmune pathogenesis of MS, which may uncover extra mechanisms of the B-cell contribution to the autoimmune effects and provide novel targets for future selective MS treatment [103].

Glatiramer acetate (GA); Copaxone; copolymer 1 exerts a clinical response in MS patients via its modulation of IFN-γ and IL-4 by reducing the expression of IFN-γ and ensuring the stable expression of IL-4 in anti-CD3/CD28-stimulated PBMCs [102]. Moreover, GA enhances the suppressive effects of Tregs in MS [104]. Studies of human DCs have shown that GA modulates the production of inflammatory mediators without affecting DC maturation or immune-stimulatory potential. DCs exposed to GA secrete low levels of the Th1-polarizing factor IL12p70 [105] and induce IL4-secreting effector Th2 cells such as IL-10 [106].

These results show that APCs, including DCs, are essential for the GA-mediated shift in Th-cell phenotypes and indicate that DCs are an important target of the immunomodulatory effects of GA.

Mitoxantrone, a cytotoxic drug with immunomodulatory properties, is used to treat progressive MS forms [107]. Mitoxantrone increases the *ex vivo* production of the Th2 cytokines IL-4 and IL-5, but with no significant changes in IFN-γ, TNF-α, IL-10, or IL-17 expression by CD4^+^ T cells, indicating that the immune-modulation afforded by mitoxantrone treatment in MS acts through the enhancement of Th2-type cytokines [108].

Currently, a head-to-head race for approval had initially developed between two under-the-spotlight oral immunomodulatory agents—fingolimod and cladribine [109].

Fingolimod (FTY720/Gilenya, Novartis), an S1PR modulator [110], is under the spotlight because it has completed phase III trials [111] and has been approved by the FDA (Food and Drug Administration) as the first oral, first-line treatment for relapsing MS [112,113]. S1PR is mainly expressed by immune cells, neuronal cells, endothelial cells, and smooth muscle cells [114–117] and have key roles in angiogenesis, neurogenesis, and the regulation of immune cell trafficking [118–120].

The immunomodulatory effect of fingolimod acts in two pathways:

- inhibits the function of S1PR, which facilitates the CC-chemokine receptor 7-(CCR7-) mediated retention of T cells in the lymph nodes, including naïve and memory T cells. In this way, it reduces the infiltration of inflammatory cells into the CNS [121,122] and reduces the numbers of autoreactive Th17 cells that are recirculating via the lymph and blood to the CNS [123–125].
- prohibits neuroinflammation via the modulation of the S1PR1 expressed on oligodendrocytes, neurons, astrocytes, and microglia [126,127].

Another oral immunomodulatory drug, cladribine (2-chlorodeoxyadenosine) (which has been withdrawn for US market for MS), is a synthetic chlorinated deoxyadenosine analog [128] that is activated by intracellular phosphorylation in specific cell types, resulting in preferential and sustained reduction of peripheral T and B cells, mimicking the immunedeficient status of hereditary adenosine deaminase deficiency [129]. Orally administered cladribine shows significantly efficacy in MS patients [130]. Oral cladribine reduces relapses by 55%–58% and has an impact on disability progression and all MRI outcome markers in patients with relaxing/remitting MS [130–132]. Nevertheless, to exactly weigh the benefits of both novel immunomodultory agents against the potential risks is necessary and must be monitored continually.

These advances in identifying unique therapeutic targets for MS have instigated numerous phase II and phase III clinical trials, for example, trials of various mAbs, including those directed against CD52 (alemtuzumab), CD25 (daclizumab), and CD20 (rituximab), and trials of disease-modifying therapies, such as teriflunomide, laquinimod, and fumarate [133]. For example, alemtuzumab targets the surface molecule CD52 on all T-cell populations and other cellular components of the immune system, such as thymocytes, B cells, and monocytes [134].

Minocycline, an oral semisynthetic tetracycline antibiotic, can penetrate the CNS and has interesting pleiotropic biological functions and neuroprotective effects, including in demyelinating diseases such as MS [135]. A study about the impact of oral minocycline on clinical and MRI outcomes and serum immune molecules during the 24 months of open-label minocycline treatment evidenced that no relapses occurred between months 6 and 24, and the levels of the p40 subunit of IL12 were elevated during the 18 months of treatment, which might have counteracted the pro-inflammatory effects of IL-12R [136].

## 5. Conclusions

Multiple sclerosis is the most common disabling CNS disease in young adults. It is characterized by recurrent relapses and/or progression, which are attributable to multifocal brain and/or spinal cord inflammation [137]. The effector Th cells and correlated cytokines, especially IL-17, play a well-recognized role in the initiation of autoimmune tissue inflammation, and have an established association with the pathogenesis of this disorder [28].

Komiyama and colleagues demonstrated that EAE was significantly suppressed in IL17−/− mice, and was manifested as delayed onset, reduced maximum severity, with ameliorated histological changes and early recovery [138]. However, the outcomes have varied when the differentiation and/or functions of Th17 cells have been blocked in clinical trials of human autoimmune diseases, with notable success only in psoriasis and Crohn’s disease, but negative results in relapsing/remitting MS. The strategy of inhibiting the Th17 response has had even less support in preclinical studies in animal models [139].

These data raise the questions of whether MS is mediated solely by Th1 cells or solely by Th17 cells, whether it is mediated by both pathways, or whether perhaps it is mediated by neither pathway [137]. There is growing evidence that autoreactive T cells (particularly Th1 and Th17 cells) participate in the MS patho-physiology. Although the exact roles of Th1 and Th17 cells in the development of MS lesions are not well understood, it appears that both these effector T-cell populations can cause CNS inflammation and demyelinating lesions in MS and EAE [140,141].

Our increasing understanding of the immunopathogenic roles of Th1, Th2, Th17 cells and Tregs in MS should facilitate the development of novel immune-modulatory therapeutic approaches to MS [142,143].

Currently approved disease-modifying treatments achieve their effects primarily by blocking the pro-inflammatory response in a nonspecific manner. Their limited clinical efficacy calls for a more differentiated and specific therapeutic approach. We can confidently say that IFN-β, GA, and mitoxantrone are fairly clinically effective for MS patients. The addition of minocycline has also shown benefits in the MS treatment. More immune-modulatory therapeutic agents are currently in clinical trials, including fingolimod (FTY720, alemtuzumab, and rituximab add-on therapies) [144]. The extensive clinical application of these possible new immune-modulatory therapeutic agents will be under close scrutiny in the near future.

In conclusion, from basic research efforts and preclinical findings in EAE models it is clear that possibilities exist for better MS treatments. The designs of simple and good clinical studies by caring neurologists, a courageous attitude by the pharmaceutical industry and political support for these new developments will be needed if we want to improve the life-quality of MS patients and reduce the social costs needed for this chronic disease. Although no prevention or cure for MS exists, patients may count on limited drug discovery successes from the past and on continued efforts to find new, more efficient and better tolerated ways of fighting this disease.

However, efficiency in drug development can be enhanced on the basis of combination therapies, whereas side effects may be decreased by better formulations and lower doses in combination therapies.

## Figures and Tables

**Figure 1:** The Remnant Epitopes Generate Autoimmunity (REGA) model. Multiple sclerosis is a multifactorial autoimmune disease of unknown etiology. Different factors (host genetics, environmental determinants, and especially the immune system) can influence the disease progression.

**Figure 2:** T helper cell differentiation. When naïve CD4+ T cells, classified by absence of CD25 and high levels of CD62L, encounter specific antigens, they can differentiate into different effector subsets. It is likely that several “master” transcription factors, individually required for T-cell differentiation towards one of the end effector stages, are initially expressed upon engagement of the TCR with costimulatory receptors. Each transcription factor drives a specific set of genes required for lineage commitment and the expression of signature cytokines and negatively affects alternative pathways. However, the microenvironment is the driving force that determines the outcome of the differentiation course. Th1 cells are established in the presence of IFN-γ and IL-12 and signaling via STAT1 and STAT4, resulting in the expression of the master transcription factor T bet. Th2 cells depend on IL-4 and STAT6 for the increased expression of GATA3, whereas the simultaneous presence of TGF-β results in the development of Th9 cells, utilizing an undefined master transcription factor. The presence of TGF-β, with IL-2 signaling via STAT5, is known to generate, at least *in vitro*, inducible Treg, which utilize Foxp3. Also, it is TGF-β in combination with IL-6 signaling via STAT3 that drives the expression of RORγt, resulting in the differentiation of Th17 cells.
